The article "Inhibition of PAD4 enhances radiosensitivity and inhibits aggressive phenotypes of nasopharyngeal carcinoma cells" was retracted in 2024. Reasons: errors in the data; unreliable results or conclusions; concerns about the data; concerns about the images.

# Inhibition of PAD4 enhances radiosensitivity and inhibits aggressive phenotypes of nasopharyngeal carcinoma cells

**DOI:** 10.1186/s11658-021-00251-2

**Published:** 2021-03-16

**Authors:** Hao Chen, Min Luo, Xiangping Wang, Ting Liang, Chaoyuan Huang, Changjie Huang, Lining Wei

**Affiliations:** 1 Department of Endoscopy, The Affiliated Tumor Hospital of Guangxi Medical University, Nanning, 530021 Guangxi China; 2 Department of Oncology, The Second Nanning People’s Hospital, No.13 Dancun Road, Jiangnan District, Nanning, 530031 Guangxi China

**Keywords:** PAD4, GSK484, Radiosensitivity, Nasopharyngeal carcinoma

## Abstract

**Background:**

Nasopharyngeal carcinoma (NPC) is a tumor deriving from nasopharyngeal epithelium. Peptidyl-arginine deiminase 4 (PAD4) is a vital mediator of histone citrullination and plays an essential role in regulating disease process. Radiotherapy is an essential method to treat NPC. In this research, we explored the effect of PAD4 on NPC radiosensitivity.

**Methods:**

We enrolled 50 NPC patients, established mice xenograft model, and purchased cell lines for this study. Statistical analysis and a series of experiments including RT-qPCR, clonogenic survival, EdU, Transwell, and wound healing assays were done.

**Results:**

Our data manifested that PAD4 (mRNA and protein) presented a high expression in NPC tissues and cells. GSK484, an inhibitor of PAD4, could inhibit activity of PAD4 in NPC cell lines. PAD4 overexpression promoted the radioresistance, survival, migration, and invasion of NPC cells, whereas treatment of GSK484 exerted inhibitory effects on radioresistance and aggressive phenotype of NPC cells. Additionally, GSK484 could attenuate the effect of PAD4 of NPC cell progression. More importantly, we found that GSK484 significantly inhibited tumor size, tumor weight and tumor volume in mice following irradiation.

**Conclusions:**

PAD4 inhibitor GSK484 attenuated the radioresistance and cellular progression in NPC.

**Supplementary Information:**

The online version contains supplementary material available at 10.1186/s11658-021-00251-2.

## Background

Recent studies have revealed that genetic factors, viral infection, and environment are main factors resulting in the occurrence of nasopharyngeal carcinoma (NPC) [1–4]. The incidence rate of NPC ranks the first in the ear, nose and throat malignant tumors in China [5], and the major factors leading to mortality are local relapse and distant metastasis [6]. The 5-year survival rate is about 10% for radiation-resistant patients and 30% for radiation-sensitive patients [7]. Radioresistance severely hampers the efficacy of radiotherapy for patients. Therefore, understanding potential mechanism of NPC radioresistance is of great significance to exploring new strategies for treatment of NPC.

Peptidyl-arginine deiminase (PAD), including five isozymes (PAD1−4 and PAD6), can catalyze the reaction of protein citrullination, a process where arginine is converted into residue citrulline [8, 9]. PAD-mediated citrullination can modify multiple cell processes through altering tertiary structure of peptide chain, protein-protein interaction, or generation of neo-epitopes [10, 11]. Protein citrullination plays a key role in mediating protein to exert various pathophysiological effects within one polypeptide chain [12, 13]. Current studies show that protein citrullination is closely related to cancer pathogenesis [14, 15]. Emerging evidence suggests that citrullinated proteins are promising biomarkers for cancer therapy [16]. PAD4 belongs to PAD family [17], converting peptidyl arginine to peptidyl citrulline [18]. The upregulation of PAD4 was reported in varied malignancies, such as rectal adenocarcinoma, breast cancer, and ovarian cancer [19]. Studies have shown that PAD4-catalyzed neutrophil extracellular trap (NET) formation is upregulated in multiple tumors [20]. Multiple components (such as matrix metalloproteinase-9, neutrophil elastase and cathepsin G) in Nets can increase cancer cell growth, angiogenesis and distant metastasis [21, 22]. PAD4 is co-expressed with cytokeratin (CK) in a variety of cancer tissues. CK 8, CK 18, and CK 19 are citrullinated by PAD4, and citrullinated CK antagonizes the cytoskeleton depolymerization process mediated by aspartic acid-specific cysteine proteolytic enzyme, thereby inhibiting tumor cell apoptosis [23]. PAD4 can also affect the metastasis and erosion of tumor cells. The interleukin-8 generated by tumor and microenvironment exerts a critical effect in cancer cell survival, migration, and invasion. PAD4 can convert arginine at the fifth position of interleukin-8 to citrulline to restrain the biological activity of citrullinated interleukin-8 [24]. The generation of tumor-associated thrombosis is related to PAD4 and is usually accompanied by hypercitrullinated levels of histones in plasma in patients with tumor-associated thrombotic microangiopathy [25]. Additionally, PAD4 inhibitors fluoramidine or chloramidine are cytotoxic to a variety of tumor cells, including breast cancer cells, leukemia cells, and colorectal cancer cells [26]. Although numerous studies reveal the essential role of PAD4 in human cancers, its role in NPC is not identified.

In this investigation, we explored the role of PAD4 and its inhibitor GSK484 in radioresistance and phenotypes of NPC cells, which demonstrates the potential of PAD4 inhibition for treatment of NPC.

## Materials and methods

### Tissue specimens

NPC tumor specimens were collected from 50 patients with NPC at the Second Nanning People’s Hospital. Informed consent was signed by every participant enrolled in this research. The Ethics Committee of the Second Nanning People’s Hospital approved this study. Approval number: 2019-055 April 9, 2019.

### Cell culture

NPC cells (C666-1, 6-10B and 5-8F) and a normal human nasopharyngeal cell line NP69 were procured from the ATCC (MA, USA). They were grown in RPMI 1640 medium (Gibco, USA) with 10% FBS (Gibco) in a humidified incubator containing 5% CO_2_ at 37 ℃. NPC cells were treated with gradient concentrations of GSK484 (0, 5, 10, and 20 µm), respectively, for 3 h.

### Cell transfection

The pcDNA3.1/PAD4 and pcDNA3.1 were synthesized by Invitrogen. 0.2 µg of vectors were transfected into NPC cells utilizing Lipofectamine 3000 (Invitrogen, USA). After 48 h, the transfection efficiency was tested by RT-qPCR. The cells subjected to transfection was treated with 10 µm GSK484 for 3 h.

### RT-qPCR

RNA from NPC tissues or cells was isolated by a TRIzol kit (Invitrogen, USA). NanoDrop (Thermo Scientific, USA) was employed for RNA quantification at an A260/A280 ratio. 1 µg RNA was reverse transcribed to cDNA by a M-MLV Reverse Transcriptase (Invitrogen). A SYBR Premix Ex Taq II Kit (Takara, Japan) was used for RT-qPCR. GAPDH served as an endogenous control for PAD4. Relative expression of PAD4 (Forward: CCCAAACAGGGGGTATCAGT; Reverse: CCACGGACAGCCAGTCAGAA) was calculated using the 2^−ΔΔCt^ method [27].

### Clonogenic survival

NPC cells were planted into 6-well plates (Shanghai Zengyou, biotechnology, Shanghai, China) (8000 cells/well) for 24 h. Next, a medical linear accelerator (Precise accelerator, Elekta, Sweden) was used to treat cells with 0, 2, 4, 6, 8 Gy X-ray irradiation at room temperature, respectively. Afterwards, cells were further incubated for 14 days and stained with 1% crystal violet (Beijing Solaibo Technology, China). The colonies over 50 cells were recorded using a light microscope (Olympus Corporation). Surviving fraction was analyzed by the formula: Surviving fraction = amount of colonies/number of total cells × seeding efficiency of the control group.

### EdU assay

The transfected C666-1 cells were inoculated in a 24-well plate (Shanghai Zengyou, biotechnology) and cultured with 50 µM of EdU reagent (RiboBio, Guangzhou, China) for 2 h. Cells were fixed with paraformaldehyde (Sigma-Aldrich), and treated with 100 µl of Apollo solution (Sigma-Aldrich) for 30 min. After that, cell nuclei were dyed by DAPI (Sigma-Aldrich) for 5 min. A fluorescence microscope (Nikon Corporation, Japan) was employed to record EdU positive cells.

### Wound healing assay

The transfected C666-1 cells were cultured in a 6-well plate (Shanghai Zengyou, biotechnology) in serum-free medium (Gibco). When the culture reached 85%, a 20 µL sterile pipette tip (Gene Era Biotech, USA) was used to scratch the cell layer. After washing, cells were incubated in 1% FBS culture medium (Gibco). After 48 h, images were obtained at different time points by a light microscope (Nikon).

### Transwell assay

Briefly, the upper chamber was pre-coated with Matrigel (BD Biosciences, USA), and then 1 × 10^4^ cells were plated in the top chamber of Transwell (Corning Life Sciences, USA) while 500 µL of RPMI 1640 medium with 20% FBS was added to the bottom chamber. After 24 h, the invaded cells were fixed with pre-cooled methanol (Sigma-Aldrich) for 5 min and stained with 1% crystal violet (Beijing Solaibo Technology) for 5 min at room temperature. Images were obtained utilizing a light microscope (magnification, ×100; Nikon).

### Xenograft mouse model

The animal study was approved by the Institutional Animal Care and Use Committee of The Second Nanning People’s Hospital. Briefly, 5-week-old BALB/C nude mice (Vital River Laboratories Co., Ltd, Beijing, China) were administrated with subcutaneous injection of 3 × 10^6^ C666-1 cells. For GSK484 in vivo treatment, mice were treated with GSK484 (4 mg/kg) or vehicle (10% DMSO in PBS) through intraperitoneal injection 1 week after tumor implantation, followed by daily dose. The tumor growth was measured using a caliper every 10 days. Tumor volume was calculated by the formula: volume = length× width^2^ × 0.5.

### Tumor radiosensitivity study

As described previously [28], mice were grouped into no irradiation group (n = 4) or irradiation group (n = 4). Irradiation was given 20 days later. Mice in each group were irradiated with 8 Gy irradiation. All mice were killed 20 days following irradiation. Then, tumors were photographed and weighed. Tumor volume was determined by the formula: V = 0.5 × longitudinal diameter × latitudinal diameter^2^.

### Statistical analysis

Statistical analysis was conducted with SPSS 20.0 software (IBM Inc., USA). Data are displayed as the mean ± SD and all experiments were repeated three times. Student’s test was employed for comparing statistics between two groups while one-way ANOVA, followed by Tukey’s post hoc test were used for comparing differences among three or more groups. p < 0.05 was statistically significant.

## Results

### PAD4 is highly expressed in NPC

First, the PAD4 level in NPC tissues was evaluated by RT-qPCR and western blot, and the data demonstrated that PAD4 was high in NPC tissues (Fig. 1a, b). Similarly, the elevated expression of PAD4 was also detected in NPC cells (C666-1, 6-10B and 5-8F) (Fig. 1c, d). Additionally, we also tested the expression levels of the other PAD isozymes (including PAD1, PAD2, and PAD3) in NPC cells, and found that these PAD isozymes had no observable expression change in NPC cells (Additional file 1: Figure S1). Therefore, we hypothesize that PAD4 is the major isozyme in NPC.

**Fig. 1:** The expression of PAD4 in NPC. **a**, **b** RT-qPCR and western blot for the PAD4 level in NPC tissues and normal tissues. Paired Student’s test. **c**, **d** RT-qPCR and western blot for the PAD4 level in NPC cells and NP69 cells. One‑way ANOVA with Tukey’s post hoc test. *p < 0.05, **p < 0.01

### PAD4 overexpression promotes the radioresistance and cellular processes in NPC

The role of PAD4 in NPC was then investigated. PAD4 expression at mRNA and protein level was significantly upregulated by pcDNA3.1/PAD4 in C666-1 and 6-10B cells (Fig. 2a, b). To probe the function of PAD4 on the radiosensitivity of NPC, we performed colony formation assay which revealed that highly expressed PAD4 significantly increased the survival fraction of NPC cells exposed to different dose of radiation (Fig. 2c). EdU assay showed that 6 Gy dose of irradiation repressed the proliferation of C666-1 cells, while overexpressed PAD4 promoted cell proliferation at 24 h after irradiation (Fig. 2d, e). Subsequently, through wound healing assay, PAD4 overexpression facilitated the migratory potential of C666-1 cells at 24 h under irradiation (Fig. 2f). Moreover, Transwell assay indicated that the invasive ability of C666-1 cell after irradiation was increased after PAD4 overexpression (Fig. 2g). Overall, overexpression of PAD4 inhibits radiosensitivity and promotes malignant character of NPC cells.

**Fig. 2:** PAD4 overexpression promotes the radioresistance and cellular processes in NPC. **a**, **b** The PAD4 level in NPC cells transfected with pcDNA3.1/PAD4 by RT-qPCR and western blot. **c** Colony formation assay for cell survival under different doses of radiation. **d**, **e** Cell proliferation in NPC cells transfected pcDNA3.1/PAD4 by EdU assay, at 24 h after 6 Gy irradiation. **f**, **g** Migration and invasion in NPC cells transfected pcDNA3.1/PAD4 by wound healing and Transwell, at 24 h after 6 Gy irradiation. Unpaired Student’s test. *p < 0.05, **p < 0.01

### Inhibition of PAD4 promotes the radiosensitivity and cellular processes in NPC

Next, different concentrations of PAD4 inhibitor (GSK484) was used to treat C666-1 and 6-10B cells. The data delineated that GSK484 concentration-dependently decreased the expression of PAD4 (Fig. 3a, b). As shown in Fig. 3b, the survival fraction of NPC cells exposed to irradiation was significantly inhibited after treatment of GSK484 (Fig. 3c). The results from EdU assay showed that treatment of GSK484 suppressed cell proliferation after irradiation (Fig. 3d). Furthermore, analysis of migration and invasion revealed that treatment of GSK484 restrained the migratory and invasive ability of C666-1 cells (Fig. 3e, f). We further detected the changes of histone citrullination (citH3) to examine whether the activity of PAD4 is in relation to treatment or no treatment with PAD4 inhibitor. Western blot demonstrated that the citH3 protein levels were markedly reduced by PAD4 inhibition (Fig. 3g). The above findings suggested that GSK484 exerts inhibitory effects on radioresistance and aggressive phenotypes of NPC cells through inhibiting the activity of PAD4.

**Fig. 3:** Inhibition of PAD4 promotes the radiosensitivity and cellular processes in NPC. **a**, **b** The PAD4 level after treatment with GSK484 by RT-qPCR and western blot. **c** Colony formation assay of NPC cells treated with different concentrations of GSK484. One‑way ANOVA with Tukey’s post hoc test. **d** Cell proliferation in NPC cells treated with GSK484 or not by EdU assay, at 24 h after 6 Gy irradiation. **e**, **f** Migration and invasion in NPC cells treated with GSK484 or not by wound healing and Transwell assays, at 24 h after 6 Gy irradiation. **g** The level of citH3 protein in NPC cell treated with GSK484 or not was measured by western lot. Unpaired Student’s test. *p < 0.05, **p < 0.01

### Treatment of GSK484 attenuates the effect of PAD4 overexpression of NPC cell progression

As observed in Fig. 4a, b, GSK484 treatment significantly downregulated the expression of PAD4 upregulated by pcDNA3.1/PAD4 in C666-1 cells. Colony formation assay demonstrated that GSK484 treatment reversed the promotive effect of PAD4 overexpression on the survival fraction of C666-1 cells (Fig. 4c). Moreover, the effects on the increase of aggressive phenotypes of C666-1 cells caused by PAD4 were abrogated after treatment of GSK484 (Fig. 4d, f). Furthermore, in Fig. 4g, citH3 was significantly elevated in PAD4 overexpressed cells but knocked down by GSK484, suggesting that histone citrullination occurs in a PAD4-dependent way. These results suggested the key role of GSK484 in inhibiting the effects of PAD4 on radiosensitivity and malignant phenotype of NPC cells.

**Fig. 4:** Treatment of GSK484 attenuates the effect of PAD4 overexpression of NPC cell functions. **a**, **b** The PAD4 level in NPC cells treated differently by RT-qPCR and western blot analyses. **c** Colony formation assay for the survival of NPC cells treated differently. **d** Cell proliferation in NPC cells treated differently by EdU assay. **e**, **f** Migration and invasion ability in NPC cells treated differently by wound healing and Transwell. **g** The citH3 protein levels in NPC cell treated differently by western lot. One‑way ANOVA with Tukey’s post hoc test. *p < 0.05, **p < 0.01

**Fig. 5:** GSK484 inhibits tumor growth and reverses radioresistance in vivo. C666-1 cells treated with 10 µm GSK484 or 0 µm GSK484 were injected into mice, n = 4, tumor growth curves (**a**), weights (**b**) and images (**c**). Unpaired Student’s test. *p < 0.05, **p < 0.01

### GSK484 inhibits tumor growth and reverses radioresistance in vivo

Since GSK484 could reverse the effect of PAD4 on radioresistance of NPC in vitro, we intended to verify whether it is applicable in vivo. Tumor grow curves revealed that the tumors grew significantly slower in mice treated with GSK484 than in the control group. Additionally, the mice treated with GSK484 were more sensitive to irradiation (Fig. 5a). The weights and images of the tumors further suggested that GSK484 significantly suppressed tumor growth after irradiation (Fig. 5b, c). Overall, GSK484 inhibits tumor growth and reverses radioresistance in vivo.

## Discussion

NPC is an epithelial malignancy with a high mortality and is a major cause of cancer-associated death in South China, North Africa, and Southeast Asia [29]. Since cancers cells are sensitive to ionizing radiation (IR), up to date, radiotherapy has become a preferred method for cancer treatment [30, 31]. NPC patients at early stage tend to be efficiently subjected to radiotherapy [32]. Additionally, radiotherapy in combination with immunotherapy or chemotherapy may affect tumor immune response, giving rise to clinical improvement in various tumors [33]. Although better tumor localization through advanced radiotherapy techniques can help improving local control of NPC, radioresistance, which may result in tumor recurrence and metastasis, is a major barrier to long-term survival [34, 35]. One and a half years after radiotherapy, most patients with NPC suffer from local recurrence and distant metastasis [34]. Thus, exploring the mechanisms of radioresistance in NPC is essential for identifying more effective therapies for NPC.

More and more reports have indicated that PAD4 was a possible gene involved in epigenetic and phenotypic alteration in various cancers [36–38]. In the present study, the upregulated mRNA and protein expression of PAD4 in NPC was demonstrated, which is in line with the previous results that PAD4 is overexpressed in a variety of malignancies [39]. Since different cancers do have different PAD isozyme dominance, we performed an assessment on this through measuring the expression of the other isozymes in NPC cells. Our data revealed that these PAD isozymes had no significant expression change in NPC cells. Therefore, we concluded that PAD4 is the major isozyme in NPC. NPC cells were transfected with stable overexpression vector of PAD4 to determine the role of PAD4 in NPC progression. Interestingly, our findings showed that upregulated PAD4 promoted malignant character of NPC cells. As reported previously, inhibition of PAD4 suppresses the invasive and migratory phenotypes of lung cancer cells [40]. Silencing PAD4 attenuates gastric cancer cell proliferation, invasion, and cell cycle [38]. PAD4 facilitates gastric tumorigenesis via enhancing the expression of several oncogenes [41]. These literatures demonstrate the oncogenic property of PAD4 in tumorigenesis.

GSK484 hydrochloride suppresses the PAD4 target protein citrullination and reduces NETs formation by binding to low-calcium form of PAD4 in a selective and reversible way [42]. GSK484 is selective for PAD4 over PAD1–3. It binds at a different site from the amidines, a conformation of the PAD4 active site where part of the site is re-ordered to form a β-hairpin [42]. To test the phenotypes of NPC cells in the absence of PAD4, we used GSK484 to treat NPC cells. As expected, GSK484 treatment of cell lines decreased the expression of PAD4 (mRNA and protein) in a concentration-dependent manner. Moreover, GSK484 markedly inhibited the malignant character of NPC cells. Previous studies proved the regulatory role of PAD4 in cancers through citrullination. PAD4-driven citrullination of a key matrix component collagen type I contributes to mesenchymal-to-epithelial transition (EMT), a phenotypic conversion that occurs in cancer cells, and liver metastasis in colorectal cancer [16]. Ectopically expressing wild type PAD4 promotes osteosarcoma cell invasion and migration while PAD4 mutation with no citrullination activity fails to affect cell phenotypes [43]. Subsequently, to examine whether this effect is associated with its citrullination activity, the changes of citH3 were detected to examine the citrullination activity of PAD4 in the context of GSK484. The results revealed treatment with GSK484 reduced the levels of citH3 protein, which is also an indicator of PAD4 activity, suggesting that GSK484 exerts inhibitory effects on NPC progression through inhibiting the citrullination activity of PAD4. However, since GSK484 is a reversible inhibitor of PAD4, prolong the incubation time between GSK484 and PAD4 may prevent the inactivation of PAD4. A deeper investigation verifying this point should be performed in the future. Interestingly, a study indicated that loss of PAD4 accelerates induction of EMT and invasion of tumors in breast cancer by the citrullination of nuclear GSK3β activating TGF-β pathway [44]. This finding is contrary to our study. The differences in cancer cell response to PAD4 may be due to the function diversity of PAD4 in different cancers.

However, there are certain limitations to our work. The mechanism by which PAD4 regulates its targets in NPC is unclear. Additionally, it is unknown whether there are other PAD isozymes or molecules such as GSK3β involved in PAD4-mediated phenotypic alternation in NPC. PAD4 has been shown to act as a transcriptional coregulator of many factors including p53, ING4, ELK1, p21, p300,and CIP1 [45–47]. Studies have indicated that the link between PAD4 and carcinogenesis is mediated through the p53 tumor suppressor gene via citrullination of citH3 [45] or the ELK1 oncogene to activate cFos [48]. Therefore, a significant future direction is to identify the potential targets or signaling pathways that PAD4 mediates in NPC.

## Conclusions

In summary, PAD4 was upregulated in NPC, and its upregulation increased the radioresistance, and cellular processes in NPC, whereas its inhibitor GSK484 elicited inhibitory effects on these phenotypes. Moreover, GSK484 significantly inhibited tumor growth in vivo. Therefore, PAD4 may be a novel biomarker for NPC treatment. Other enzymes or molecules may participate in the PAD4-mediated NPC progression and further investigation could be done in the future.

## Supplementary Information

**Additional file 1: Figure S1. **The expression level of the other PAD isozymes in NPC. RT-qPCR for the expression of PAD1 (A), PAD2 (B), and PAD3 (C) in NPC cell lines and NP69 cells. One‑way ANOVA with Tukey’s post hoc test.

## Data Availability

All data from this study are available in this published article.

## Abbreviations

NPC: Nasopharyngeal carcinoma
PAD4: Peptidyl-arginine deiminase 4

## References

[1] Liu D, Wang Y, Zhao Y, Gu X (2020). LncRNA SNHG5 promotes nasopharyngeal carcinoma progression by regulating miR-1179/HMGB3 axis. BMC Cancer.

[2] Vaughan TL, Shapiro JA, Burt RD, Swanson GM, Berwick M, Lynch CF (1996). Nasopharyngeal cancer in a low-risk population: defining risk factors by histological type. Cancer Epidemiol Biomark Prev.

[3] Chua MLK, Wee JTS, Hui EP, Chan ATC (2016). Nasopharyngeal carcinoma. Lancet.

[4] He XS, Deng M, Yang S, Xiao ZQ, Luo Q, He ZM (2008). The tumor supressor function of STGC3 and its reduced expression in nasopharyngeal carcinoma. Cell Mol Biol Lett.

[5] Wei KR, Zheng RS, Zhang SW, Liang ZH, Li ZM, Chen WQ (2017). Nasopharyngeal carcinoma incidence and mortality in China, 2013. Chin J Cancer.

[6] Kim YS, Kim BS, Jung SL, Lee YS, Kim MS, Sun DI (2008). Radiation therapy combined with (or without) cisplatin-based chemotherapy for patients with nasopharyngeal cancer: 15-years experience of a single institution in Korea. Cancer Res Treat.

[7] Bruce JP, Yip K, Bratman SV, Ito E, Liu FF (2015). Nasopharyngeal cancer: molecular landscape. J Clin Oncol.

[8] Bicker KL, Thompson PR (2013). The protein arginine deiminases: structure, function, inhibition, and disease. Biopolymers.

[9] Asaga H, Ishigami A (2007). Microglial expression of peptidylarginine deiminase 2 in the prenatal rat brain. Cell Mol Biol Lett.

[10] Vossenaar ER, Zendman AJ, van Venrooij WJ, Pruijn GJ (2003). PAD, a growing family of citrullinating enzymes: genes, features and involvement in disease. BioEssays.

[11] Witalison EE, Thompson PR, Hofseth LJ (2015). Protein arginine deiminases and associated citrullination: physiological functions and diseases associated with dysregulation. Curr Drug Targets.

[12] Henderson B, Martin AC (2014). Protein moonlighting: a new factor in biology and medicine. Biochem Soc Trans.

[13] Jeffery CJ (2018). Protein moonlighting: what is it, and why is it important?. Philos Trans R Soc Lond Ser B Biol Sci.

[14] Yuzhalin AE (2019). Citrullination in cancer. Cancer Res.

[15] Mohanan S, Cherrington BD, Horibata S, McElwee JL, Thompson PR, Coonrod SA (2012). Potential role of peptidylarginine deiminase enzymes and protein citrullination in cancer pathogenesis. Biochem Res Int.

[16] Yuzhalin AE, Gordon-Weeks AN, Tognoli ML, Jones K, Markelc B, Konietzny R (2018). Colorectal cancer liver metastatic growth depends on PAD4-driven citrullination of the extracellular matrix. Nat Commun.

[17] Anzilotti C, Pratesi F, Tommasi C, Migliorini P (2010). Peptidylarginine deiminase 4 and citrullination in health and disease. Autoimmun rev.

[18] Nakashima K, Hagiwara T, Ishigami A, Nagata S, Asaga H, Kuramoto M (1999). Molecular characterization of peptidylarginine deiminase in HL-60 cells induced by retinoic acid and 1alpha,25-dihydroxyvitamin D(3). J Biol Chem.

[19] Chang X, Han J (2006). Expression of peptidylarginine deiminase type 4 (PAD4) in various tumors. Mol Carcinog.

[20] Erpenbeck L, Schön MP (2017). Neutrophil extracellular traps: protagonists of cancer progression?. Oncogene.

[21] Zhang Q, Li J, Liu F, Li Z, Comments on Li H (2015). A systematic review of matrix metalloproteinase 9 as a biomarker of survival in patients with osteosarcoma. Tumour Biol.

[22] Houghton AM, Rzymkiewicz DM, Ji H, Gregory AD, Egea EE, Metz HE (2010). Neutrophil elastase-mediated degradation of IRS-1 accelerates lung tumor growth. Nat Med.

[23] Chang X, Han J, Pang L, Zhao Y, Yang Y, Shen Z (2009). Increased PADI4 expression in blood and tissues of patients with malignant tumors. BMC Cancer.

[24] Nierodzik ML, Karpatkin S (2006). Thrombin induces tumor growth, metastasis, and angiogenesis: Evidence for a thrombin-regulated dormant tumor phenotype. Cancer Cell.

[25] Demers M, Wagner DD (2014). NETosis: a new factor in tumor progression and cancer-associated thrombosis. Semin Thromb Hemost.

[26] Slack JL, Causey CP, Thompson PR (2011). Protein arginine deiminase 4: a target for an epigenetic cancer therapy. Cell Mol Life Sci.

[27] Livak KJ, Schmittgen TD (2001). Analysis of relative gene expression data using real-time quantitative PCR and the 2(-Delta Delta C(T)) Method. Methods.

[28] Shen L, Xia M, Deng X, Ke Q, Zhang C, Peng F (2020). A lectin-based glycomic approach identifies FUT8 as a driver of radioresistance in oesophageal squamous cell carcinoma. Cell Oncol.

[29] Tang LL, Chen WQ, Xue WQ, He YQ, Zheng RS, Zeng YX (2016). Global trends in incidence and mortality of nasopharyngeal carcinoma. Cancer Lett.

[30] Jagsi R (2014). Progress and controversies: radiation therapy for invasive breast cancer. Cancer J Clin.

[31] He Y, Jing Y, Wei F, Tang Y, Yang L, Luo J (2018). Long non-coding RNA PVT1 predicts poor prognosis and induces radioresistance by regulating DNA repair and cell apoptosis in nasopharyngeal carcinoma. Cell Death Dis.

[32] Peng H, Chen L, Chen YP, Li WF, Tang LL, Lin AH (2018). The current status of clinical trials focusing on nasopharyngeal carcinoma: A comprehensive analysis of ClinicalTrials.gov database. PLoS ONE.

[33] Rekers NH, Troost EG, Zegers CM, Germeraad WT, Dubois LJ, Lambin P (2014). Stereotactic ablative body radiotherapy combined with immunotherapy: present status and future perspectives. Cancer Radiother.

[34] Lee AW, Poon YF, Foo W, Law SC, Cheung FK, Chan DK (1992). Retrospective analysis of 5037 patients with nasopharyngeal carcinoma treated during 1976–1985: overall survival and patterns of failure. Int J Radiat Oncol Biol Phys.

[35] Kristensen CA, Kjaer-Kristoffersen F, Sapru W, Berthelsen AK, Loft A, Specht L (2007). Nasopharyngeal carcinoma. Treatment planning with IMRT and 3D conformal radiotherapy. Acta Oncol (Stockholm Sweden).

[36] Kolodziej S, Kuvardina ON, Oellerich T, Herglotz J, Backert I, Kohrs N (2014). PADI4 acts as a coactivator of Tal1 by counteracting repressive histone arginine methylation. Nat Commun.

[37] Christophorou MA, Castelo-Branco G, Halley-Stott RP, Oliveira CS, Loos R, Radzisheuskaya A (2014). Citrullination regulates pluripotency and histone H1 binding to chromatin. Nature.

[38] Xin J, Song X (2016). Role of peptidylarginine deiminase type 4 in gastric cancer. Exp Ther Med.

[39] Chang X, Fang K (2010). PADI4 and tumourigenesis. Cancer Cell Int.

[40] Liu M, Qu Y, Teng X, Xing Y, Li D, Li C (2019). PADI4-mediated epithelial–mesenchymal transition in lung cancer cells. Mol Med Rep.

[41] Zheng Y, Zhao G, Xu B, Liu C, Li C, Zhang X (2016). PADI4 has genetic susceptibility to gastric carcinoma and upregulates CXCR2, KRT14 and TNF-α expression levels. Oncotarget.

[42] Lewis HD, Liddle J, Coote JE, Atkinson SJ, Barker MD, Bax BD (2015). Inhibition of PAD4 activity is sufficient to disrupt mouse and human NET formation. Nat Chem Biol.

[43] Zhai Q, Qin J, Jin X, Sun X, Wang L, Du W (2020). PADI4 modulates the invasion and migration of osteosarcoma cells by down-regulation of epithelial-mesenchymal transition. Life Sci.

[44] Stadler SC, Vincent CT, Fedorov VD, Patsialou A, Cherrington BD, Wakshlag JJ (2013). Dysregulation of PAD4-mediated citrullination of nuclear GSK3β activates TGF-β signaling and induces epithelial-to-mesenchymal transition in breast cancer cells. Proc Natl Acad Sci USA.

[45] Tanikawa C, Ueda K, Nakagawa H, Yoshida N, Nakamura Y, Matsuda K (2009). Regulation of protein Citrullination through p53/PADI4 network in DNA damage response. Cancer Res.

[46] Yao H, Li P, Venters BJ, Zheng S, Thompson PR, Pugh BF (2008). Histone Arg modifications and p53 regulate the expression of OKL38, a mediator of apoptosis. J Biol Chem.

[47] Guo Q, Fast W (2011). Citrullination of inhibitor of growth 4 (ING4) by peptidylarginine deminase 4 (PAD4) disrupts the interaction between ING4 and p53. J Biol Chem.

[48] Zhang X, Gamble MJ, Stadler S, Cherrington BD, Causey CP, Thompson PR (2011). Genome-wide analysis reveals PADI4 cooperates with Elk-1 to activate c-Fos expression in breast cancer cells. PLoS Genet.

